This article has been retracted.

# Exogenous Hydrogen Sulfide Mitigates Oxidative Stress and Mitochondrial Damages Induced by Polystyrene Microplastics in Osteoblastic Cells of Mice

**DOI:** 10.1155/2023/2516472

**Published:** 2023-02-18

**Authors:** Qingping Shi, Feihong Chen, Yuanyi Feng, Yangxi Zheng, Ximei Zhi, Wen Wu

**Affiliations:** ^1^The Second School of Clinical Medicine, Southern Medical University, Guangzhou, Guangdong 510515, China; ^2^Department of Endocrinology, Guangdong Geriatrics Institute, Guangdong Provincial People's Hospital, Guangdong Academy of Medical Sciences, Guangzhou, Guangdong 510080, China; ^3^Department of Geriatric Medicine, People's Hospital of Shenzhen Baoan District, Affiliated Hospital of Shenzhen Bao'an of Southern Medical University, The Second Affiliated Hospital of Shenzhen University, Shenzhen, Guangdong 518000, China; ^4^Department of Respiratory Medicine, People's Hospital of Shenzhen Baoan District, Affiliated Hospital of Shenzhen Bao'an of Southern Medical University, The Second Affiliated Hospital of Shenzhen University, Shenzhen, Guangdong 518000, China

## Abstract

Polystyrene microplastics (mic-PS) have become harmful pollutants that attracted substantial attention about their potential toxicity. Hydrogen sulfide (H_2_S) is the third reported endogenous gas transmitter with protective functions on numerous physiologic responses. Nevertheless, the roles for mic-PS on skeletal systems in mammals and the protective effects of exogenous H_2_S are still indistinct. Here, the proliferation of MC3T3-E1 cell was analyzed by CCK8. Gene changes between the control and mic-PS treatment groups were analyzed by RNA-seq. The mRNA expression of bone morphogenetic protein 4 (Bmp4), alpha cardiac muscle 1 (Actc1), and myosin heavy polypeptide 6 (Myh6) was analyzed by QPCR. ROS level was analyzed by 2′,7′-dichlorofluorescein (DCFH-DA). The mitochondrial membrane potential (MMP) was analyzed by Rh123. Our results indicated after exposure for 24 h, 100 mg/L mic-PS induced considerable cytotoxicity in the osteoblastic cells of mice. There were 147 differentially expressed genes (DEGs) including 103 downregulated genes and 44 upregulated genes in the mic-PS-treated group versus the control. The related signaling pathways were oxidative stress, energy metabolism, bone formation, and osteoblast differentiation. The results indicate that exogenous H_2_S may relieve mic-PS toxicity by altering *Bmp4*, *Actc1*, and *Myh6* mRNA expressions associated with mitochondrial oxidative stress. Taken together, this study demonstrated that the bone toxicity effects of mic-PS along with exogenous H_2_S have protective function in mic-PS-mediated oxidative damage and mitochondrial dysfunction in osteoblastic cells of mice.

## 1. Introduction

Polystyrene microplastics (mic-PS) are plastic particles with diameter < 5 mm [1], originating from industrial products and plastics demoted into pieces by UV radiation, physical, or biodegradation [2]. Mic-PS contain high-density and low-density polyethylene (HD/LD-PE), polyethylene terephthalate (PET), polypropylene (PP), and polyvinylchloride (PVC), together with polystyrene microplastic (PS-MP) [3]. More recently, these minor plastic products have been widely detected in freshwater organisms, ranging from algae to fish, even in mammals. Therefore, pollution by mic-PS was classified as the second most crucial threat in ecological environment at the United Nations Environmental Conference in 2015 [4].

Mic-PS less than 20 *μ*m can easily access the mammalian tissues, while mic-PS with particle size of 0.1~10 *μ*m can effectively pass through the cytomembrane, intestinal mucosal barrier, and blood-brain barrier, even transmit through the placenta to the next generation [5, 6]. Further investigation substantiates the toxicity of mic-PS on index such as oxidative stress, enzymatic activity, quantity of egg laying, feeding rate, and growth rate [5–7]. Specific polystyrene mic-PS with size of 5 to 20 *μ*m can accrue in the liver, lung, and kidney; additionally, they can evoke oxidative damage along with metabolic alterations [8, 9]. In contrast, it remains unknown the relationship among mic-PS intake and bone destruction of terrestrial mammals.

Hydrogen sulfide (H_2_S), a colorless indispensable endogenous gas, can subsequently enhance catalytic activity by attaching hydropersulfide group (-SSH) to relevant cysteine residues into targeted protein. Exogenous H_2_S has been reported to regulate numerous signaling pathways associated with biological processes, for instance, regulation of kinase, maintaining intracellular mitochondrial ATP generation, and scavenging reactive oxygen species (ROS). In osteoblastic cell, the scavenging ability to reduce oxidative stress and sustaining maintenance of mitochondrial membrane potential is a key signal for cells and is a crucial target of osteoporosis responsible for increased bone fracture threat. Further research on mic-PS stated that exogenous H_2_S increases the expression of heme oxygenase-1 and NAD(P)H : quinone oxidoreductase 1, consequently decreasing microplastics producing hepatic apoptosis and inflammation [10]. Therefore, exogenous H_2_S might be an innovative antioxidant medium under MP stress system. So far, the beneficial effect of exogenous H_2_S in mic-PS-induced bone toxicity remains undiscovered.

In this study, we aimed to study the cytotoxic effects of mic-PS in MC3T3-E1 cells, then investigating the toxicity of mic-PS in osteoblastic cell through RNA sequencing (RNA-seq). Finally, we aimed to explore whether H_2_S ameliorated mic-PS exposure induced damage by attenuating oxidative stress and mitochondrial damage.

## 2. Materials and Methods

### 2.1. Materials and Reagents

Mic-PS (100 nm) were purchased from the Tianjin DAE Scientific Co. Ltd (Tianjin, China). GYY4137 (as the donor of H_2_S) and rhodamine 123 (Rh123) were bought from Sigma (St. Louis, MO, USA). 2′,7′-Dichlorofluorescein diacetate (DCFH-DA) was obtained from Nanjing Jiancheng Bioengineering Institute (Nanjing, China). Cell counting kit-8 (CCK-8) was obtained from Dojindo Laboratories (Kumamoto, Japan). Fetal bovine serum (FBS) and Gibco minimum essential medium *α* (*α*-MEM) were purchased from Thermo Fisher (Waltham, MA, USA).

### 2.2. Cell Culture and Treatment

The mouse calvaria-derived MC3T3-E1 osteoblasts were bought commercially from the National Collection of Authenticated Cell Cultures (Shanghai, China). Osteoblasts were seeded at 1 × 10^5^ cells/mL into 75 cm^2^ flasks, cultured in *α*-MEM supplemented with FBS (10%). The basic medium was replaced every three days. The growing conditions were at 37°C with 5% CO_2_. There were four groups, including the control group, mic-PS group, mic-PS+H_2_S group, and H_2_S group. The concentration of H_2_S released from GYY4137 was 100 *μ*M.

### 2.3. Cell Viability Assay

MC3T3-E1 cells (1 × 10^4^ cells/ml) were cultured in 96-well plates. Then they were incubated for 24 hours at 37°C. The cells were washed with phosphate-buffered saline (PBS), and the cell counting kit-8 (10 *μ*l, at 10% dilution) was added in each well. After incubation, the absorbance was measured with the Multiskan MK3 microplate reader (Thermo Fisher). The mean optical density (OD) was conducted to count the cell viability (%) following the equation (OD_treatment_/OD_control_) × 100. The cell viability assay in each group was repeated five times.

### 2.4. Measurement of Intracellular ROS Generation

MC3T3-E1 cells were incubated with 10 *μ* M of 2′,7′-dichlorofluorescein (DCFH-DA) for 30 minutes at 37°C. Then, the cells were washed with PBS. The DCF fluorescence was visualized through a fluorescence microscope. The mean fluorescence intensity (MFI) indicated the amount of ROS in the intracellular environment. The measurements were performed by using the ImageJ software (version 1.8.0, Bethesda, Maryland, USA). The experiment was performed three times.

### 2.5. Examination of the Mitochondrial Membrane Potential (MMP)

The MC3T3-E1 cells were incubated for 45 minutes at 37°C with Rh123 (2 *μ*M). Then, the cells were washed with PBS. The fluorescence was then detected by a fluorescence microscope. The MFI of five random fields indicated the levels of MMP. The measurements were performed by using the ImageJ software (version 1.8.0).

### 2.6. mRNA Library Construction and Sequencing

The total RNA was isolated, purified, and next quantified by the NanoDrop ND-1000 spectrophotometer (Thermo Fisher Scientific, USA). The RNA integrity was assessed by Bioanalyzer 2100 (Agilent Technologies, CA) and later confirmed by gel electrophoresis. After purification from the total RNA (1 *μ*g) with Dynabeads Oligo (dT)_25_ (Thermo Fisher), the poly(A) RNA was fragmented through the Magnesium RNA Fragmentation Module (NEB, Ipswich, MA, USA). Then, the cleaved fragments were reverse transcribed through the SuperScript Reverse Transcriptase (Invitrogen, USA) and used to synthetize U-labeled, second-stranded DNA. The AMPure XP bead was used to perform the size selection. Later, the ligated products were expanded through the polymerase chain reaction (PCR). The denaturation was initially performed for 3 minutes at 95°C. Then, 8 cycles of denaturation were performed for 15 seconds at 98°C. The annealing was performed for 15 seconds at 60°C, with a following extension for 30 seconds at 72°C. The final extension was conducted at 72°C for 5 minutes. Regarding the final cDNA library, the average insert size was 300 ± 50 bp. The 2 × 150 bp paired-end sequencing (PE150) was done with the NovaSeq 6000 sequencing system (Illumina).

### 2.7. Quantitative Real-Time PCR (QPCR) Analysis

The total RNA of MC3T3-E1 cells was extracted and amplified using a SYBR Green based real-time PCR assay (Eppendorf, Germany). The PCR reaction was performed holding for 3 minutes at 95°C, then for 10 seconds at 95°C, for 30 seconds at 60°C, and for further 35 seconds at 72°C. The comparative cross threshold method was used to quantify the mRNA expression. The QPCR in each group was repeated three times. For primer sequences, see Table 1.

### 2.8. Statistical Analysis

Continuous variables are described as mean ± standard error of the mean (SEM). Comparisons were tested by one-way analysis of variance (ANOVA) followed by Dunnett's test using GraphPad Prism 8.0.2 software. A *p* < 0.05 was considered statistically significant.

## 3. Results

### 3.1. Cytotoxic Effects of Mic-PS in MC3T3-E1 Cells

To evaluate the cytotoxic effects of mic-PS in MC3T3-E1 cells, we treated the cells with different times and concentrations. As shown in Figure 1(a), MC3T3-E1 cells were exposed to increasing concentrations of mic-PS with the same 24 hours. Mic-PS at 50 mg/L showed no significant effects on cell viability (*p* > 0.05). Mic-PS at 100 and 150 mg/L displayed toxic effects on MC3T3-E1 cells (*p* < 0.01), with no statistical difference between the two concentrations (*p* > 0.05). Remarkably, both concentrations lead to a decline in cell viability to almost 50% compared to the control group (*p* < 0.01). Therefore, mic-PS at 100 mg/L was used in the following time-response experiment (Figure 1(b)). Exposed MC3T3-E1 cells to mic-PS for 24 hours and 36 hours induced considerable cytotoxicity; the maximum decrease in cell viability was observed at 24 h (*p* < 0.01). In accordance with the above results, the MC3T3-E1 cells were cultured with mic-PS at 100 mg/L for 24 h in the following experiments.

### 3.2. Mic-PS Treatment Induced Gene Expression Change in MC3T3-E1 Cells

Next, to further investigate the different gene expressions that occur between the mic-PS and control groups, RNA-seq was conducted. There were 147 differentially expressed genes (DEGs) (absolute Log2 fold change ≥ 1, *p* ≤ 0.05). Among them, 103 genes were downregulated, while 44 genes were upregulated (Figure 1(c)). The top 100 genes with the lowest *p* value were further evaluated by hierarchical clustering analysis (Figure 1(d)). This analysis showed a clear distinction between the mic-PS and control groups.

### 3.3. The Gene Ontology (GO) Enrichment Analysis and Kyoto Encyclopedia of Genes and Genomes (KEGG) Enrichment Analysis

GO biological process (GO-BP), GO cellular component (GO-CC), and GO molecular function (GO-MF) were the three sections of the GO enrichment analysis (Figure 2(a)). According to the three parts of the GO analysis, the upregulated and downregulated DEGs were functionally categorized, especially regulation of transcription, inflammatory response, protein binding, oxidation-reduction process, and apoptotic. A biological pathway distribution was observed in KEGG enrichment analysis between the mic-PS and control groups (Figure 2(b)). There were several signaling pathways influenced by mic-PS, including peroxisome proliferator-activated receptors (PPAR), arginine and proline metabolism, thyroid hormone metabolism, estrogen metabolism, cyclic adenosine monophosphate (cAMP), phosphonate and phosphinate metabolism, and calcium signal transduction pathway. The signaling pathways are probably related to oxidative stress resistance, energy metabolism, osteoblast differentiation, and bone formation. Thus, the regulated oxidative stress resistance and mitochondrial ATP energy metabolism might be the determinative mechanism linking mic-PS to dysfunction in MC3T3-E1 cells.

### 3.4. Exogenous H_2_S Reduced Mic-PS-Induced Cytotoxicity in MC3T3-E1 Cells

As described in Figure 3(a), exposure of MC3T3-E1 cells to 100 mg/L mic-PS for 24 hours induced considerable cytotoxicity (*p* < 0.01). When cells were treated with H_2_S at 100 *μ*M, 24 hours, they are markedly ameliorated from mic-PS injury (*p* < 0.01). We evaluated the effects of H_2_S and mic-PS on ROS levels in MC3T3-E1 cells. As expected, mic-PS elevated ROS levels, but the effect was reversed by H_2_S (*p* < 0.01) (Figures 3(b) and 3(g)). Similar findings were obtained with the MMP. The mic-PS exposure reduced MMP (*p* < 0.01). On the contrary, H_2_S treatment alleviated (*p* < 0.01) the reduced MMP mediated by mic-PS (Figures 3(c) and 3(h)). The above results revealed that exogenous H_2_S inhibits mic-PS-induced cytotoxicity, oxidative stress, and dissipation of MMP damage.

### 3.5. Exogenous H_2_S Increased the Mitochondrial Damage-Related Gene Expression

According to the bioinformatic analysis and above results, we chose bone morphogenetic protein 4 (*Bmp4*), alpha cardiac muscle 1 (*Actc1*), and myosin heavy polypeptide 6 (*Myh6*) as the potential candidate genes. To verify whether these three genes are involved in H_2_S signaling pathway, mRNA expression was tested by QPCR. Expression of these three gene expressions decreased in the mic-PS group, while exogenous H_2_S increased a certain extent of these three genes (*p* < 0.01, Figures 3(d)–3(f)). Besides, we observed that mic-PS treatment most affected the Actc1 gene expression, while the effect of mic-PS on *Bmp4* expression was comparable minimal. These results suggested that H_2_S increases *Bmp4*, *Actc1*, and *Myh6* expressions to mitigate mic-PS-induced oxidative stress and mitochondrial damage in osteoblastic cell.

## 4. Discussion

Since the durability and indecomposable features of plastics as discarded pollutants, the plastic contaminants have risen dramatically worldwide. 322 million tons were produced in 2015 [11], while it will increase by 33 billion tons in 2050 as predicted [12]. Mic-PS can be detected everywhere, including human biological samples. Thus, it is meaningful to study the toxicity of mic-PS in mammals. Previous data have shown that mic-PS induces intestinal microbial growth, reproductive toxicity, metabolic disorders, and intestinal barrier dysfunction in mice [13, 14]. Nevertheless, little is known about mic-PS effects on mouse bone metabolism. In this study, we found that mouse osteoblastic cell activity declined after being exposed to mic-PS. RNA-seq analysis showed 147 differentially expressed genes between the mic-PS and control groups. Furthermore, we proved that exogenous H_2_S could increase the related gene expression to reduce mic-PS-induced oxidative stress and mitochondrial injury (Figure 4).

The bioinformatic analysis was subsequently performed to evaluate the toxicity of mic-PS in mouse osteoblastic cell through GO and KEGG databases. GO analysis indicates that exposure to mic-PS significantly affected biological processes such as transcription, inflammatory response, protein binding, oxidation-reduction process, and apoptotic. Currently studies suggest that inducing oxidative stress was the relevant effect of mic-PS toxicity [15, 16]. Xu et al. researched on human lung epithelial cells; they proved that mic-PS significantly affect the cell viability via inducing significant upregulation of proinflammatory and proapoptotic proteins, including TNF-*α*, IL-8, caspase-3, caspase-8, and caspase-9 [17]. Based on the KEGG databases in our study, involving peroxisome proliferator-activated receptors (PPAR), arginine and proline metabolism, thyroid hormone, estrogen, cyclic adenosine monophosphate(cAMP), phosphonate and phosphinate metabolism, and calcium pathway were significantly enriched pathways for DEGs. PPAR signaling pathway was also observed in exposure to MPs on grass carp through KEGG enrichment analysis [18]. PPARs are transcription factors that regulate the expression of genes involved in energy and lipid metabolism; it is interesting that activation of PPAR*δ* improves mitochondrial function [19]. Presently, Sun et al. reported that Jak/Stat pathway, nicotinamide metabolism, and unsaturated fatty acids are associated with mic-PS-mediated toxicity in the mouse hematological system; furthermore, they found that decreased Nnt is possibly correlated with reduced antioxidant power and mitochondrial damage after mic-PS exposure [20]. Oxidative stress and mitochondrial metabolic changes are closely related to osteogenic capacity. Mitochondrial dysfunction and ROS rise induced osteoblast senescence and osteoblast activity [21] and led to type 2 diabetic osteoporosis [22]. Proanthocyanidins and notoginsenoside R1 treatments reduced ROS level and weakened mitochondrial dysfunction to improve osteoblast activity [23, 24]. These studies suggest that oxidative stress and disturbances in mitochondrial metabolism are targets for improving osteogenic capacity. Hence, the change of oxidative stress and mitochondrial metabolism was selected for further toxicity mechanism caused by exposure to mic-PS in this research.

To validate of the potential of the change of oxidative stress and mitochondrial metabolism after mic-PS exposure, we then performed experiments in vitro. The mic-PS exposure significantly elevated oxidative stress, as well as dissipated MMP, while exogenous H_2_S mitigated mic-PS-induced oxidative and mitochondrial injury. Presently, accumulating evidence has demonstrated that Bmp4, Actc1, and Myh6 are closely related to homeostasis of mitochondria and redox reactions [25–27]. Especially, BMP4 is a group of bone growth factors firstly identified because of their capability to enhance bone and cartilage formation. As a result, these three genes (*Bmp4*, *Actc1*, and *Myh6*) were selected. We next used QPCR to test our findings. We observed that the downward trend of QPCR results in the mic-PS group was essentially comparable with the sequencing analysis. A similar alteration of *Bmp4* and *Myh5* had also been observed in zebrafish exposed to mic-PS (100 *μ*g/L) [28]. However, Bhagat et al. described upregulation of bmp4 in zebrafish embryos when exposed to polystyrene nanoplastics (1 mg/L) and azole fungicides (ketoconazole and fluconazole) [29]. Different size and concentration of mic-PS should be considered in making the results. Meanwhile, experimental results of Umamaheswari et al. indicated that mic-PS exposure upregulated the gstp1, hsp70l, and ptgs2a gene expressions, while it downregulated cat, sod1, gpx1a, and ache genes, illustrating the potential of mic-PS to mediate different degrees of toxic effects in aquatic animals through changing ROS medicated oxidative stress altering its metabolic process, histological architecture, and gene regulatory modes [30].

Of note, in a range of biological mechanisms, exogenous H_2_S has essential physiological and pathological impacts. According to a recent study, exogenous H_2_S protects osteoblastic cells from H_2_O_2_-induced cell oxidative stress injury [31]. In this study, the findings supported the inhibitory effect of exogenous H_2_S on mic-PS-induced mitochondrial damage and oxidative stress in mouse osteoblastic cells. In addition, exogenous H_2_S considerably increases the alleviated expression of *Bmp4*, *Actc1*, and *Myh6* derived from mic-PS. The mechanisms underlying mic-PS-induced oxidative stress and mitochondrial damage could be complex and diverse. Mic-PS has been shown to reduce the activity of glutathione S-transferases, limiting detoxification and resulting in ROS generation [32]. Moreover, it is generally acknowledged that H_2_S is associated with increasing glutathione S-transferase transcript level. Recently, a study has demonstrated that H_2_S suppressed inflammation and oxidative stress induced by mic-PS in mouse liver via upregulated Keap1-Nrf2 pathway [10]. Notably, *Bmp4*, *Actc1*, and *Myh6* were reported to be associated with glutathione S-transferases. Reportedly, exogenous H_2_S improved the *BMP4* expression in rat pulmonary arterial smooth muscle cells [33]. Thus, these results indicate that exogenous H_2_S may relieve mic-PS toxicity by altering *Bmp4*, *Actc1*, and *Myh6* expressions associated with mitochondrial oxidative stress.

The study has two main limitations. First, the effect of exogenous H_2_S and mic-PS needs to be explored in vivo. Second, the downstream signaling pathways regulated by H_2_S in mic-PS-induced injury need to find in further exploration.

## 5. Conclusion

In conclusion, we used RNA-seq and validation experiment at molecular and cellular levels to demonstrate that mic-PS (100 mg/L) caused a significant toxicity in osteoblastic cells in mice (an advanced mammal), while exogenous H_2_S may considerably mitigate mic-PS-induced oxidative stress and mitochondrial damage through increasing *Bmp4*, *Actc1*, and *Myh6* expressions. Our research unveiled the bone toxicity effects of mic-PS and provides novel insights in the mechanism of exogenous H_2_S protective function in mic-PS-induced bone injury.

## Figures and Tables

**Figure 1:** Cytotoxic effects of mic-PS in MC3T3-E1 cells. (a) Increasing concentrations (50, 100, and 150 mg/L) of mic-PS were added to MC3T3-E1 cells for 24 hours seeded in 96-well plate. (b) MC3T3-E1 cells were cultured with 100 mg/L mic-PS with different times. Continuous variables are displayed as mean ± standard error of the mean (*n* = 5) (^∗∗^*p* < 0.01 vs. control group). (c) Volcano plot visualizing the statistical difference of the DEGs. (d) Heatmap displaying the genes with the lowest *p* value.

**Figure 2:** GO enrichment analysis and KEGG enrichment analysis. (a) GO terms significantly enriched in DGEs of mic-PS vs. control (*p* < 0.05). (b) KEGG analyses showed top twenty regulated pathways in MC3T3-E1 cells with 100 mg/L mic-PS compared to control group. *p* values were shown through different color. The sizes of the bubble indicate the gene count for each pathway.

**Figure 3:** Exogenous 100 *μ*M H_2_S reduced 100 mg/L mic-PS-induced toxicity in MC3T3-E1 cells. (a) Cell viability evaluated through the CCK-8 assay. (b) Quantitative analysis for the MFI of DCFH-DA in different groups. (c) Quantitative analysis for the MFIs of Rh123 in different groups. (d–f) Expression of different mRNAs in different groups was tested by QPCR. (d) *Bmp*4, (e) Actc1, and (f) *Myh*6. (g, h) Representative fluorescent photographs of assessing the intracellular ROS/MMP level in different groups. (g) ROS and (h) MMP. Continuous variables are displayed as mean ± standard error of the mean (*n* = 5). ^∗∗^*p* < 0.01. Scale bar: 100 *μ*m.

**Figure 4:** Proposed mechanistic schematic diagram of H_2_S mitigates mic-PS-induced oxidative stress and mitochondrial damage in mouse osteoblastic cell.

**Table 1:** Sequences of primers used for the QPCR assay.

Gene	Primer sequences (5′ to 3′)
GAPDH	Forward: GAGAAACCTGCCAAGTATGATGAC
	Reverse: TAGCCGTATTCATTGTCATACCAG

Bmp4	Forward: CAACTCAACCAACCATGCCATTGTG
	Reverse: TTCAACACCACCTTGTCATACTCATCC

Myh6	Forward: TGGCACCGTGGACTACAACATTATG
	Reverse: CAGCAGAAGCATAGGTAGAGAAGAGTG

Actc1	Forward: GACTCTCTTCCAGCCCTCTTTCATTG
	Reverse: GGTGCCTCCAGATAGGACATTGTTG

## Data Availability

The research data are available upon request.

## Supplementary Materials

Supplementary 1 Table S1: data used for CCK8 with different concentrations of mic-PS.

Supplementary 2 Table S2: data used for CCK8 with different times of mic-PS.

Supplementary 3 Table S3: data used for CCK8/ROS/MMP.

Supplementary 4 Table S4: data used for QPCR analysis.
